# Perception of the Use of the Direct Observation of Procedural Skills in Occupational Therapy Postgraduate Year Training in Taiwan: Survey of the Perspectives of Trainees and Supervisors

**DOI:** 10.1155/2023/8013086

**Published:** 2023-05-24

**Authors:** Yi-chia Liu, Yi-chen Lee, Pai-chuan Huang, I-Hui Lee, Keh-chung Lin

**Affiliations:** ^1^Department of Psychiatry, National Cheng Kung University Hospital, College of Medicine, National Cheng Kung University, Tainan, Taiwan; ^2^Department of Occupational Therapy, College of Medicine, National Cheng Kung University, Tainan, Taiwan; ^3^School of Occupational Therapy, College of Medicine, National Taiwan University, Taipei, Taiwan; ^4^Graduate Institute of Early Intervention, College of Medicine, Chang Gung University, Taoyuan, Taiwan; ^5^Department of Psychiatry, College of Medicine, National Cheng Kung University, Tainan, Taiwan; ^6^Division of Occupational Therapy, Department of Physical Medicine and Rehabilitation, National Taiwan University Hospital, Taipei, Taiwan

## Abstract

**Introduction:**

Assessment of clinical competence is a significant part of the training for young occupational therapists (OTs). Objective and systematic assessment allows both supervisors and trainees to be aware of the training objectives and monitor the progress. The direct observation of procedural skills (DOPS) is a work-based assessment to evaluate professional knowledge, skills, and attitude in clinical training. This study investigated the perspectives of OT educators and trainees on using DOPS and their discrepancy for OT postgraduate year (PGY) training.

**Methods:**

This study used a quantitative online survey. Eighty-six supervisors and 41 trainees of OT PGY training programs from 95 hospitals returned the questionnaire (a 90.5% return rate), and 64 supervisors and 30 trainees who used DOPS were analyzed. Outcomes included the practicality in using the DOPS in clinical settings, the ease of rating the DOPS, and advantages and the disadvantages of the DOPS.

**Results:**

Most respondents reported that completing one DOPS required at least 11 minutes for direct observation (11-40 minutes: teacher 92.2%; trainee 80.6%). Most respondents (teacher 96.9%, trainee 96.8%) had feedback after direct observation of DOPS, and about half of the feedback assessments took 5 to 10 minutes (teacher 53.1%, trainee 48.4%). Most OT educators and trainees agreed that clinical resources were sufficient and that DOPS matched with OT training goals, benefited OT competence training, and had a fair, objective, and consistent scoring system. Significantly higher percentages of OT trainees felt stressed in and satisfied with the DOPS assessment than trainers. Differences between teachers and trainees regarding easiness of rating DOPS items were not significant.

**Conclusion:**

Most OT educators and trainees agreed that DOPS was a practical and appropriate assessment for OT PGY training.

## 1. Literature Review

Clinical education is the most important part of health professional education [1] and also one of the strategies for developing continuing competence in occupational therapy (OT) [2]. The postgraduate year (PGY) training program for general medicine was implemented by the Taiwanese government in 2003 [3] and for other health care professions in 2007, including OT [4], pharmacy [5], and nursing [6], to address a need for improved professional training and the quality of health care services. The programs are implemented by the Joint Commission of Taiwan under the supervision and instruction of the relevant professional associations to equip PGY trainees with (1) professional knowledge, the ability to provide quality care, evidence-based skills, and resource management ability; (2) patient-centered, comprehensive, and holistic perspectives and skills; (3) professional ethical reasoning and communication skills; and (4) the ability to work in a team [7, 8].

Assessment of clinical competence is a significant part of the training for young OTs. Objective and systematic assessment allows both supervisors and trainees to be aware of the training objectives and monitor the progress. The assessment of practical performance in clinical conditions (does) is ranked as the highest level in Miller's hierarchical model for the assessment of clinical competence [9]. Direct observation of procedural skills (DOPS) is a workplace-based assessment tool specifically designed to assess practical skills. It requires the assessor to directly observe a trainee conducting a procedure, document the evaluation in a checklist, and give feedback to the trainee based on objective findings [10].

Several studies have reported the experiences of supervisors and trainees with the DOPS in health professional training, such as medical, nursing, and veterinary students, and showed that examiners and examinees were both very satisfied with the DOPS [10, 11]. However, the feasibility and user experience of the DOPS for OT PGY training has not been examined. We investigated the perception of OT supervisors and trainees on the DOPS in Taiwan for PGY training. Therefore, the aims of our study were to investigate (1) the experience of using the DOPS in clinical settings, (2) the ease of rating clinical performance with the DOPS, and (3) the advantages and disadvantages of the DOPS for OT PGY training.

## 2. Methods

### 2.1. Procedures

This is a cross-sectional survey study. Data were collected from January 2017 to December 2018. We invited the teaching directors of each hospital to participate in this project from January 2017 to June 2017. A link to the online questionnaire was sent from July 2017 to December 2017. As of January 2018, the response rate was not good. The second recruitment and first reminder were carried out from January 2018 to July 2018. Follow-up reminders were sent one and two months later. Information in the database of the Ministry of Health and Welfare, Taiwan, was used to invite OT chiefs in charge of OT PGY training programs in 2017 to participate in this study. The online questionnaire was sent by email along with regular postal mail to participants. Participants signed an informed consent to be included in this study, and their data coding and analysis were anonymized. In our first part of the electronic questionnaire, there was the background of the questionnaire, the purpose of the research, the use of data, and the informed consent form. After downloading the filled forms, any identified information was removed, and then the deidentified data were used for data coding and analysis. When the online electronic questionnaire URL was given, each respondent was asked to report a unique user number to be used while filing the survey, which was convenient for distinguishing the source and avoiding repeated collection of operations.

### 2.2. Instrument

Prior to using DOPS for assessment, training included a 2 hours of general introduction to DOPS and a 2-hour scoring consistency workshop. This questionnaire was developed by two senior OTs (Y. C. Liu and P. C. Huang) based on the research questions and literature of medical education with work-based assessment in 2015 [11–14]. Five experts in OT PGY training were invited to assess and discuss the questionnaire in a focus group, and revised this questionnaire accordingly. A second group of five external experts in OT fieldwork education and research were invited to revise and finalize the questionnaire.

The final questionnaire had four sections. The first section included 11 items of basic sociodemographic information of the participants, including job position, age, sex, highest educational level, teaching/working years, specialty area, status of hospital, and service location. The second section used a 5-point Likert scale to rate 21 items related to experiences with using DOPS (i.e., practicality, subjective opinion, cover domain, and scoring system). The third section assessed trainer's and trainee's perception of ease of using the DOPS in rating the clinical performance of PGY OT trainees with a 5-point Likert scale of 11 items. The fourth part included 16 items of the advantages and disadvantages of the DOPS for the evaluation of OT PGY trainees.

### 2.3. Statistical Analyses

Demographic characteristics and distribution of participants' responses in perception of DOPS are presented with descriptive statistics (i.e., frequency and percentage and mean and standard deviation). Comparisons between supervisors and trainees in experience of using DOPS, ease of rating the DOPS, and advantages and disadvantages of DOPS were assessed with the *χ*^2^ and *t* tests. Data were analyzed with SPSS 18.0 software (SPSS, Chicago, IL, USA).

## 3. Results

Completed questionnaires were returned by 86 supervisors and 41 trainees of the 95 hospitals (individuals) who received the invitational letter and survey by emails and regular mail for a 90.5% return rate. The response rate was the number of questionnaires returned divided by the number of that have applied for PGY teaching hospitals times 100%. Data from 64 supervisors and 30 trainees who had used the DOPS and completed surveys were included in the analysis. 37.2% of the participants were located in the northwestern Taiwan, 12.8% of the participants were located in the middle western Taiwan, 43.7% of the participants were located in the southwestern Taiwan, and 6.4% of the participants were located in the eastern Taiwan. The distribution of location of participants represents the population of OT in Taiwan. The demographic characteristics of the participants are presented in Table 1. Significantly more women, being younger, and lower levels of education were noted in the trainee group than in the supervisor group. There were no differences in specialty areas and classification of hospital in the two groups.

Most respondents reported that completing one DOPS required at least 11 minutes for direct observation (11-20 minutes: teacher 26.6% (*n* = 17) trainee 29.0% (*n* = 9); 21-30 minutes: teacher 34.4% (*n* = 22), trainee 38.7% (*n* = 12); 31-40 minutes: teacher 15.6% (*n* = 10), trainee 12.9% (*n* = 4)). Most respondents (teacher 96.9% (*n* = 62), trainee 96.8% (*n* = 30)) had feedback after direct observation of DOPS, and about half of the feedback assessments took 5 to 10 minutes (teacher 53.1% (*n* = 34), trainee 48.4% (n =15)). There were no differences in time for direction observation (*χ*^2^(7) = 2.29, *p* = .94) and for feedback (*χ*^2^(5) = 8.87, *p* = .11) between teachers and trainees.

The percentage of trainees who received DOPS training was 70% (*n* = 21) compared with 56.3% (*n* = 36) for teachers, which was significantly higher (*χ*^2^(2) = 16.27, *p* < .0001). There was no significant difference (*χ*^2^(3) = 4.12, *p* = .25) in terms of discussion of DOPS rating criteria among teachers before formal assessment between teachers (75%, *n* = 48) and trainees (90%, *n* = 27).

Regarding experience with DOPS, more than 70% of trainees (range: 72.4% to 93.3%) and supervisors (range: 71.3% to 85.9%) responded “strongly agree” or “agree” with most items except for teacher's rating of sufficient teachers (67.2%), assessing clinical reasoning ability (62.6%), consistency in scoring standard (61.0%), and both teachers' and trainees' rating of stressfulness in assessment (17.2% and 41.4%, respectively) and needing further training (54.7% and 55.1%, respectively). In addition, less than 10% of trainees (range: 0 to 6.8%) and supervisors (range: 0 to 9.4%) reported “strongly disagree” or “disagree” with most items except for teachers' rating of need further training (20.6%) and both trainees' and teachers' rating of stressfulness in assessment (10.3% and 23.5%, respectively). The use experience of DOPS of the trainees and supervisors and their comparisons are presented in Table 2.

Results of the *χ*^2^ tests indicated that there were significant differences between trainees and teachers on most items of experiences of using the DOPS for OT PGY training except for items of low cost, better than traditional teaching assessment, fairness, objectiveness, and consistency in scoring standard. Significantly higher percentages of “strongly agree” were noted in trainee's perception (range: 20.7% to 41.4%) than in supervisor's perception (range: 1.6% to 12.5%).

Most respondents reported “simple” (trainee range: 10.7% to 34.5%; teacher range: 23.0% to 35.0%) or “neutral” (trainee range: 17.2% to 53.6%; teacher range: 27.9% to 47.5%) in the easiness of rating most of the DOPS in clinical settings. Results of *χ*^2^ tests indicated there were no significant differences between trainees and teachers on all items of easiness of rating DOPS for OT PGY training program. The easiness of rating DOPS as reported by the trainees and supervisors and their comparisons are presented in Table 3.

The advantages of the DOPS assessment tool were ranked as follows: direct observation of clinical performance (trainee: 96.6%, supervisor: 96.8%), immediacy of feedback (trainee: 75.0%, supervisor: 76.2%), flexibility (trainee: 75.9%, supervisor: 76.2%), finishing assessment in a short period of time (trainee: 69.0%, supervisor: 69.8%), no additional funding or resource burden (trainee: 62.1, supervisor: 55.6%), and no space restriction (trainee: 58.6%, supervisor: 55.6%). Having a valid and reliable scoring system may be an issue for DOPS in the assessment of clinical competence in OT PGY training because more than 75% of respondents reported subjectivity as one of the disadvantages. The results of the *χ*^2^ tests revealed no significant differences on perceptions in advantages and the disadvantages of DOPS between trainees and supervisors.  Table 4 presents the comparison of advantages and disadvantages between trainees and supervisors.

## 4. Discussion

To the best of our knowledge, this is one of the few studies to examine the feasibility of the DOPS and explore the use experience, advantages, and disadvantages of the OT PGY training programs by including the perspectives of both trainees and supervisors. The results found that the DOPS tool was a practical measurement tool to assess the competence of OT PGY trainees.

Time for implementing DOPS and providing feedback is a significant factor for feasibility and acceptability [11]. Some studies [15, 16] found a lack of time or being seen as an additional workload in administrating the DOPS and giving feedback in physician training. This may reflect busy the clinical hours of the physicians and time constraints for using the DOPS in the clinical training of medical doctors. In contrast to findings of the above studies [11, 15, 16], approximately 90% of the respondents in this study spent at least 11 minutes for rating DOPS, and half of the respondents reported to have at least 6 to 10 minutes for feedback. Most of the trainees (86.7% agree or strongly agree) and supervisors (75% agree or strongly agree) agreed time for implementation of DOPS was sufficient for OT PCY training. In addition, more than 75% of trainees and supervisors agree that immediate feedback was one of the advantages of using DOPS in OT PGY training.

Training of rating DOPS is another significant issue for consideration in the assessment for OT PGY training. Half of the trainees (55.1%) and supervisors (54.7%) claimed that they need further training in using DOPS. Proper implementation is one of the significant factors related to the educational impacts of administrating DOPS [17] and relies on sufficient training in using assessment tools such as DOPS.

Approximately 40% of supervisors (35.9% neutral, 1.6% disagree, and 1.6% strongly disagree) did not support consistency in the scoring standard for rating DOPS in this study. Intercase variation may affect the reliability [11]. Training is needed not only on the procedure of administrating DOPS but also on scoring training on different patients or conditions. In addition, a study suggested rating of trainees' performance by at least three supervisors observing at least two procedures each to achieve good reliability [11].

Consistent with previous studies [10, 11], some trainees (41.4% agree or strongly agree) felt that taking DOPS is a stressful experience. However, the trainee's satisfaction with DOPS is high and even higher than the supervisor's. It is possible that attending a work-based examination such as the DOPS is stressful, but the trainees appreciate this experience as learning and positive although stressful experience.

### 4.1. Implications for Occupational Therapy Education

The DOPS is a practical assessment tool for OT PGY training to monitor the trainee's knowledge, skill, and attitude. Sufficient time for examination and feedback with DOPS is an essential component for successful implementation. Training for using DOPS is needed not only for the implementation procedure but also for scoring criteria across patients and conditions.

### 4.2. Strengths and Limitations

The strength of this survey included a nationally representative sample and a high response rate (more than 90%). Participants included OTs from different areas of Taiwan, clinical specialty areas of OT, and hospital settings.

The limitations included the following. This study recruited one trainer who was the major supervisor of the trainee during the period of study from each hospital. Other therapists who had once been supervisors before the study period only were excluded. Selection bias might exist. The experience of using the DOPS might be subject to recall bias because this survey was not filled out immediately after any specific DOPS assessment.

### 4.3. Future Study

In addition to trainees and supervisors in the OT PGY training programs, the DOPS is also used for the fieldwork education of senior OT students and their clinical supervisors. Future studies may investigate the user experiences of the senior OT students and their clinical supervisors in fieldwork education.

## 5. Conclusion

Most OT educators and trainees agreed that the DOPS is a practical and appropriate assessment for the OT PGY training. Sufficient time for rating the DOPS and feedback about performance is essential to learning effects. Training in using the DOPS is necessary and should include rating criteria with different conditions and patients with the same procedures.

## Figures and Tables

**Table 1:** Demographic characteristics of survey participants.

		Training teacher (*n* = 64)		Trainee (*n* = 30)		*χ* ^2^ (df)	*p*
		Frequency	Percentage	Frequency	Percentage		
Sex	Male	28	43.8%	7	23.3%	3.64 (1)	.06
	Female	36	56.3%	23	76.6%		

Age	20-25 years	0	0	23	76.7%	71.84 (4)	<.001
	26-30 years	11	17.2%	6	20.0%		
	31-35 years	14	21.9%	1	3.3%		
	36-45 years	25	39.1%	0	0		
	Over 46 years	14	21.9%	0	0		

Education	Junior college	0	0	2	6.7%	11.62 (2)	.003
	University	36	56.3%	24	80.0%		
	Master and above	28	43.8%	4	13.3%		

Teaching years	Less than 5 years	12	18.8%				
	6-10 years	19	29.7%				
	11-15 years	14	21.9%				
	16-20 years	11	17.2%				
	More than 20 years	8	12.5%				

Specialty area	Physical	21	32.8%	7	23.3%	2.74 (3)	.43
	Pediatric	3	4.7%	0	0		
	Physical and pediatric	21	32.8%	13	43.3%		
	Mental health	19	29.7%	10	33.3%		

Hospital	Medical center	20	31.3%	11	36.7%	.90 (3)	.82
	Regional teaching hospital	29	45.3%	14	46.7%		
	District teaching hospital	10	15.6%	4	13.3%		
	Psychiatric teaching hospital	5	7.8%	1	3.3%		

**Table 2:** Comparison between teachers and trainees in their rating for practicality.

Questionnaire items		Strongly agree	Agree	Neutral	Disagree	Strongly disagree	*χ* ^2^ (df)
Used at predictable time	Teacher (*n* = 64)	6 (9.4%)	45 (70.3%)	13 (20.3%)	0	0	15.23 (3)^∗∗^
	Trainee (*n* = 30)	12 (40.0%)	14 (46.7%)	3 (10.0%)	1 (3.3%)	0	
Sufficient observation time	Teacher (*n* = 64)	5 (7.8%)	43 (67.2%)	14 (21.9%)	2 (3.1%)	0	12.56 (3)^∗∗^
	Trainee (*n* = 30)	11 (36.7%)	15 (50.0%)	3 (10.0%)	1 (3.3%)	0	
Immediacy of feedback	Teacher (*n* = 64)	8 (12.5%)	44 (68.8%)	12 (18.8%)	0	0	12.68 (3)^∗∗^
	Trainee (*n* = 29)	12 (41.4%)	13 (44.8%)	3 (10.3%)	1 (3.4%)	0	
Sufficient feedback time	Teacher (*n* = 63)	6 (9.5%)	39 (61.9%)	17 (27.0%)	1 (1.6%)	0	11.46 (3)^∗∗^
	Trainee (*n* = 29)	10 (34.5%)	16 (55.2%)	2 (6.9%)	1 (3.4%)	0	
Good cooperation among supervisors, trainees, and peers	Teacher (*n* = 63)	6 (9.5%)	40 (63.5%)	16 (25.4%)	1 (1.6%)	0	10.07 (3)^∗^
	Trainee (*n* = 29)	10 (34.5%)	15 (51.7%)	3 (10.3%)	1 (3.4%)	0	
Sufficient teachers	Teacher (*n* = 64)	5 (7.8%)	38 (59.4%)	18 (28.1%)	3 (4.7%)	0	10.73 (3)^∗^
	Trainee (*n* = 29)	10 (34.5%)	11 (37.9%)	7 (24.1%)	1 (3.4%)	0	
Stressfulness in assessment	Teacher (*n* = 64)	1 (1.6%)	10 (15.6%)	38 (59.4%)	12 (18.8%)	3 (4.7%)	12.67 (4)^∗^
	Trainee (*n* = 29)	6 (20.7%)	6 (20.7%)	14 (48.3%)	3 (10.3%)	0	
Assess the trainee's learning status	Teacher (*n* = 63)	4 (6.3%)	41 (65.1%)	16 (25.4%)	2 (3.2%)	0	8.03 (3)^∗^
	Trainee (*n* = 29)	8 (27.6%)	15 (51.7%)	5 (17.2%)	1 (3.4%)	0	
Low cost	Teacher (*n* = 64)	9 (14.1%)	40 (62.5%)	14 (21.9%)	0	1 (1.6%)	6.81 (4)
	Trainee (*n* = 29)	9 (31.0%)	13 (44.8%)	5 (17.2%)	1 (3.4%)	1 (3.4%)	
Overall implementability	Teacher (*n* = 64)	7 (10.9%)	47 (73.4%)	10 (15.6%)	0	0	8.27 (3)^∗^
	Trainee (*n* = 29)	9 (31.0%)	16 (55.2%)	3 (10.3%)	1 (3.4%)	0	
Familiar with the DOPS	Teacher (*n* = 64)	6 (9.4%)	39 (60.9%)	17 (26.6%)	1 (1.6%)	1 (1.6%)	11.83 (4)^∗^
	Trainee (*n* = 30)	10 (33.3%)	18 (60.0%)	2 (6.7%)	0	0	
Need further training	Teacher (*n* = 64)	4 (6.3%)	31 (48.4%)	23 (35.9%)	5 (7.8%)	1 (1.6%)	11.39 (4)^∗^
	Trainee (*n* = 29)	7 (24.1%)	9 (31.0%)	7 (24.1%)	3 (10.3%)	3 (10.3%)	
Better than traditional teaching assessment	Teacher (*n* = 63)	8 (12.7%)	39 (61.9%)	14 (22.2%)	2 (3.2%)	0	7.22 (3)
	Trainee (*n* = 29)	9 (31.0%)	18 (62.1%)	2 (6.9%)	0	0	
Use as a teaching assessment tool	Teacher (*n* = 64)	8 (12.5%)	47 (73.4%)	9 (14.1%)	0	0	6.49 (2)^∗^
	Trainee (*n* = 29)	10 (34.5%)	17 (58.6%)	2 (6.9%)	0	0	
Matching with OT's training goals	Teacher (*n* = 64)	4 (6.3%)	42 (65.6%)	17 (26.6%)	0	1 (1.6%)	11.01 (3)^∗^
	Trainee (*n* = 29)	9 (31.0%)	16 (55.2%)	4 (13.8%)	0	0	
Assessing clinical/communication skills	Teacher (*n* = 64)	6 (9.4%)	44 (68.8%)	13 (20.3%)	1 (1.6%)	0	8.89 (3)^∗^
	Trainee (*n* = 28)	9 (32.1%)	17 (60.7%)	2 (7.1%)	0	0	
Assessing clinical reasoning ability	Teacher (*n* = 64)	4 (6.3%)	36 (56.3%)	19 (29.7%)	5 (7.8%)	0	11.37 (3)^∗^
	Trainee (*n* = 29)	8 (27.6%)	17 (58.6%)	4 (13.8%)	0	0	
Assessing standard procedural ability	Teacher (*n* = 64)	7 (10.9%)	44 (68.8%)	11 (17.2%)	2 (3.1%)	0	10.28 (3)^∗^
	Trainee (*n* = 29)	11 (37.9%)	13 (44.8%)	5 (17.2%)	0	0	
Fairness	Teacher (*n* = 64)	5 (7.8%)	42 (65.6%)	16 (25.0%)	1 (1.6%)	0	5.26 (3)
	Trainee (*n* = 29)	7 (24.1%)	17 (58.6%)	5 (17.2%)	0	0	
Objectiveness	Teacher (*n* = 64)	5 (7.8%)	41 (64.1%)	17 (26.6%)	1 (1.6%)	0	3.06 (3)
	Trainee (*n* = 29)	5 (17.2%)	19 (65.5%)	5 (17.2%)	0	0	
Consistency in scoring standard	Teacher (*n* = 64)	3 (4.7%)	36 (56.3%)	23 (35.9%)	1 (1.6%)	1 (1.6%)	7.05 (4)
	Trainee (*n* = 29)	6 (20.7%)	16 (55.2%)	7 (24.1%)	0	0	

^∗^ *p* < .05; ^∗∗^*p* < .01.

**Table 3:** Comparison between teachers and trainees in the easiness of rating the DOPS in clinical settings.

Questionnaire items		Very simple	Simple	Neutral	Difficult	Very difficult	*χ* ^2^ (df)
Demonstrates understanding of indications, relevant anatomy, and technique of procedure	Teacher (*n* = 59)	11 (18.6%)	15 (25.4%)	20 (33.9%)	10 (16.9%)	3 (5.1%)	2.05 (4)
	Trainee (*n* = 29)	3 (10.3%)	7 (24.1%)	10 (34.5%)	8 (27.6%)	1 (3.4%)	
Obtains informed consent	Teacher (*n* = 61)	27 (44.3%)	15 (24.6%)	17 (27.9%)	1 (1.6%)	1 (1.6%)	6.15 (4)
	Trainee (*n* = 29)	11 (37.9%)	8 (27.6%)	5 (17.2%)	3 (10.3%)	2 (6.9%)	
Demonstrates appropriate preparation pre-procedure	Teacher (*n* = 60)	11 (18.3%)	21 (35.0%)	21 (35.0%)	5 (8.3%)	2 (3.3%)	1.56 (4)
	Trainee (*n* = 29)	5 (17.2%)	10 (34.5%)	10 (34.5%)	4 (13.8%)	0	
Appropriate analgesia or safe sedation	Teacher (*n* = 57)	8 (14.0%)	14 (24.6%)	25 (43.9%)	6 (10.5%)	4 (7.0%)	1.53 (4)
	Trainee (*n* = 28)	3 (10.7%)	8 (28.6%)	11 (39.3%)	5 (17.9%)	1 (3.6%)	
Technical ability	Teacher (*n* = 61)	2 (3.3%)	17 (27.9%)	24 (39.3%)	16 (26.2%)	2 (3.3%)	2.60 (4)
	Trainee (*n* = 28)	1 (3.6%)	5 (17.9%)	15 (53.6%)	7 (25.0%)	0	
Aseptic technique	Teacher (*n* = 59)	14 (23.7%)	16 (27.1%)	21 (35.6%)	5 (8.5%)	3 (5.1%)	4.39 (4)
	Trainee (*n* = 28)	10 (35.7%)	4 (14.3%)	10 (35.7%)	4 (14.3%)	0	
Seeks help where appropriate	Teacher (*n* = 60)	3 (5.0%)	14 (23.3%)	27 (45.0%)	14 (23.3%)	2 (3.3%)	7.22 (4)
	Trainee (*n* = 28)	6 (21.4%)	5 (17.9%)	9 (32.1%)	8 (28.6%)	0	
Post procedure management plan	Teacher (*n* = 61)	4 (6.6%)	14 (23.0%)	25 (41.0%)	15 (24.6%)	3 (4.9%)	2.68 (4)
	Trainee (*n* = 28)	1 (3.6%)	3 (10.7%)	15 (53.6%)	8 (28.6%)	1 (3.6%)	
Communications skills	Teacher (*n* = 59)	8 (13.6%)	14 (23.7%)	22 (37.3%)	13 (22.0%)	2 (3.4%)	1.73 (4)
	Trainee (*n* = 28)	3 (10.7%)	4 (14.3%)	11 (39.3%)	9 (32.1%)	1 (3.6%)	
Consideration for patient/professionalism	Teacher (*n* = 60)	5 (8.3%)	15 (25.0%)	23 (38.3%)	12 (20.0%)	5 (8.3%)	1.42 (4)
	Trainee (*n* = 28)	4 (14.3%)	6 (21.4%)	11 (39.3%)	6 (21.4%)	1 (3.6%)	
Overall clinical competence performing procedure	Teacher (*n* = 59)	3 (5.1%)	16 (27.1%)	28 (47.5%)	12 (20.3%)	0	6.91 (4)
	Trainee (*n* = 28)	2 (7.1%)	3 (10.7%)	14 (50.0%)	7 (25.0%)	2 (7.1%)	

**Table 4:** Advantages and disadvantages of DOPS reported by trainees and supervisors.

Advantages		Yes	No	*χ* ^2^ (df)
Direct observation of clinical performance	Trainees (*n* = 29)	28 (96.6%)	1 (3.4%)	.95 (1)
	Supervisors (*n* = 63)	61 (96.8%)	2 (3.2%)	
No space restriction	Trainees (*n* = 29)	17 (58.6%)	12 (41.4%)	.78 (1)
	Supervisors (*n* = 63)	35 (55.6%)	28 (44.4%)	
Finishing assessment in a short period of time	Trainees (*n* = 29)	20 (69.0%)	9 (31.0%)	.93 (1)
	Supervisors (*n* = 63)	44 (69.8%)	19 (30.2%)	
Flexibility	Trainees (*n* = 29)	22 (75.9%)	7 (24.1%)	.97 (1)
	Supervisors (*n* = 63)	48 (76.2%)	15 (23.8%)	
Consistent scoring criteria among supervisors	Trainees (*n* = 29)	14 (48.3%)	15 (51.7%)	.13 (1)
	Supervisors (*n* = 63)	41 (65.1%)	22 (34.9%)	
Consistent scoring criteria among OT and other health care professionals	Trainees (*n* = 29)	10 (34.5%)	19 (65.5%)	.91 (1)
	Supervisors (*n* = 63)	21 (33.3%)	42 (66.7%)	
Immediacy of feedbacks	Trainees (*n* = 29)	22 (75.9%)	7 (24.1%)	.97 (1)
	Supervisors (*n* = 63)	48 (76.2%)	15 (23.8%)	
Reliable and valid rating of clinical performance	Trainees (*n* = 29)	14 (48.3%)	15 (51.7%)	.73 (1)
	Supervisors (*n* = 63)	28 (44.4%)	35 (55.6%)	
No additional funding or resource burden	Trainees (*n* = 29)	18 (62.1%)	11 (37.9%)	.56 (1)
	Supervisors (*n* = 63)	35 (55.6%)	28 (44.4%)	
Disadvantages		Yes	No	
Assessing only parts of clinical skills	Trainees (*n* = 29)	5 (17.2%)	24 (82.8%)	.08 (1)
	Supervisors (*n* = 63)	22 (34.9%)	41 (65.1%)	
Subjectivity	Trainees (*n* = 29)	22 (75.9%)	7 (24.1%)	.11 (1)
	Supervisors (*n* = 63)	56 (88.9%)	7 (11.1%)	
Low patient acceptance	Trainees (*n* = 29)	4 (13.8%)	25 (86.2%)	.95 (1)
	Supervisors (*n* = 63)	9 (14.3%)	54 (85.7%)	
Not adaptable to greater variability of clinical situations	Trainees (*n* = 29)	16 (55.2%)	13 (44.8%)	.70 (1)
	Supervisors (*n* = 63)	32 (50.8%)	31 (49.2%)	
Time restriction in clinical setting	Trainees (*n* = 29)	3 (10.3%)	26 (89.7%)	.70 (1)
	Supervisors (*n* = 63)	5 (7.9%)	58 (92.1%)	

## Data Availability

The data sets generated and analyzed during the present study are not publicly available due to participant confidentiality but are available from the corresponding author on reasonable request.

## Abbreviations

OT: Occupational therapy
DOPS: Direct observation of procedural skills
PGY: Postgraduate year.
